This article has been retracted.

# Comparative Immunogenicity of HIV-1 gp160, gp140 and gp120 Expressed by Live Attenuated Newcastle Disease Virus Vector

**DOI:** 10.1371/journal.pone.0078521

**Published:** 2013-10-01

**Authors:** Sunil K. Khattar, Sweety Samal, Celia C. LaBranche, David C. Montefiori, Peter L. Collins, Siba K. Samal

**Affiliations:** 1 Virginia-Maryland Regional College of Veterinary Medicine, University of Maryland, College Park, Maryland, United States of America; 2 Division of Surgical Sciences, Duke University, Durham, North Carolina, United States of America; 3 Laboratory of Infectious Diseases, National Institute of Allergy and Infectious Diseases, Bethesda, Maryland, United States of America; University of Delhi, India

## Abstract

The development of a vaccine against human immunodeficiency virus-1 (HIV-1) capable of inducing broad humoral and cellular responses at both the systemic and mucosal levels will be critical for combating the global AIDS epidemic. We previously demonstrated the ability of Newcastle disease virus (NDV) as a vaccine vector to express oligomeric Env protein gp160 and induce potent humoral and mucosal immune responses. In the present study, we used NDV vaccine strain LaSota as a vector to compare the biochemical and immunogenic properties of vector-expressed gp160, gp120, and two versions of gp140 (a derivative of gp160 made by deleting the transmembrane and cytoplasmic domains), namely: gp140L, which contained the complete membrane-proximal external region (MPER), and gp140S, which lacks the distal half of MPER. We show that, similar to gp160, NDV-expressed gp140S and gp120, but not gp140L, formed higher-order oligomers that retained recognition by conformationally sensitive monoclonal antibodies. Immunization of guinea pigs by the intranasal route with rLaSota/gp140S resulted in significantly greater systemic and mucosal antibody responses compared to the other recombinants. Immunization with rLaSota/140S, rLaSota/140L rLaSota/120 resulted in mixed Th1/Th2 immune responses as compared to Th1-biased immune responses induced by rLaSota/160. Importantly, rLaSota/gp140S induced neutralizing antibody responses to homologous HIV-1 strain BaL.26 and laboratory adapted HIV-1 strain MN.3 that were stronger than those elicited by the other NDV recombinants. Additionally, rLaSota/gp140S induced greater CD4+ and CD8+ T-cell responses in mice. These studies illustrate that rLaSota/gp140S is a promising vaccine candidate to elicit potent mucosal, humoral and cellular immune responses to the HIV-1 Env protein.

## Introduction

The HIV-1 envelope (Env) glycoprotein is the major viral neutralization antigen and its efficacy in protection against HIV-1 has been demonstrated in animal models [1-3]. . The HIV-1 Env also is a target for cell mediated immune responses that can contribute to protection [4,5]. Env is synthesized as a 160-kDa precursor gp160 that is processed by furin or related host cellular proteases into its soluble attachment subunit gp120 and transmembrane subunit gp41 [6,7]. gp120 and gp41 are organized on virions as trimeric spikes with three gp120 proteins non-covalently associated with three gp41 subunits [8]. The viral envelope initiates infection by contact through a gp120-CD4 interaction. This interaction also stabilizes the structure of a coreceptor binding site on gp120 that engages one of two coreceptors (CCR5 or CXCR4) [9]. The viral spike possesses a number of characteristics that subvert humoral immunity, including heavy glycosylation, conformational flexibility, and sequence variability in immunodominant domains. Therefore, significant efforts have been made to design and construct either purified Env glycoprotein immunogens or vaccine vectors that present Env glycoprotein as functional trimeric complexes, thereby preferentially exposing relevant neutralizing determinants to the immune system [10,11].

Various forms of Env glycoprotein have been evaluated as vaccine immunogens to protect against HIV-1. Env vaccines consisting of gp120 subunit proteins or peptide fragments thereof have shown a lack of protective efficacy in clinical trials [12]. Soluble forms, called gp140, which contains the membrane proximal external region (MPER) but lacks the transmembrane and cytoplasmic domains have been designed and are cleaved in the same fashion as gp160, resulting in gp120 subunits along with a thermodynamically favored 6-helix bundle formed by gp41 moiety [13-17]. Various strategies have been used to produce stable trimers of gp140 [11,18,19]. Several replication-competent and non-replication-competent viral vector have been used to express oligomeric Env immunogens and to stimulate immune responses against HIV-1 [10]. Although immunogenicity studies with these trimers have thus far showed some improvements in breadth and potency of neutralization when compared with monomeric gp120, adequate protection against diverse primary HIV-1 isolates has not been achieved.

Newcastle disease virus (NDV) is a member of the genus *Avulavirus* in the family *Paramyxoviridae*. The genome of NDV is a single-stranded, negative-sense RNA of 15 kb that contains six genes in the order 3′-N-P-M-F-HN-L-5′. [20]. NDV has several properties that are useful as a vaccine vector in humans. NDV is an avian virus that is attenuated in humans due to a natural host range restriction [21]. NDV shares only a low level of amino acid sequence identity with, and is antigenically distinct from, common animal and human pathogens, and thus vaccination should not be affected by preexisting immunity. NDV has been used to express protective antigens of several human pathogens in non-human primate models [21-24]. Further, the ability of NDV to express HIV-1 Gag [25,26] and gp160 [27] antigens and to generate Gag-and Env-specific immune response in mice and guinea pigs, respectively has been demonstrated. In the present study, we constructed NDV vectors expressing several engineered derivatives of gp160, including two forms of gp140. These were evaluated for neutralizing immune responses in guinea pigs and T-cell responses in mice. This showed that engineering gp140 containing MPER resulted in substantial increases in the induction of HIV-1-specific serum and mucosal antibodies and CD4+ and CD8+ T lymphocytes.

## Materials and Methods

### Ethical Statement

Female Hartley guinea pigs (aged 5-6 weeks) and female BALB/c mice (aged 5 weeks) were obtained from Charles River Laboratories, Wilmington, MA and National Cancer Institute, Bethesda, MD, respectively. The study was done in AAALAC-approved animal facility and under the authority of Institutional Animal Care and Use Committee (IACUC) of University of Maryland, College Park, MD. All the guinea pigs used in this study were housed in isolator cages in our Bio Safety Level-2+ facility and all the mice used in this study were kept under specific pathogen-free conditions in Individually Ventilated Cages (IVCs) in our Bio Safety Level-2+ facility. All the animals were cared for in strict accordance with established guidelines, and the experimental procedures were performed with approval from IACUC. The intranasal inoculation and bleeding in guinea pigs was performed after injecting Ketamine and Xylazine anesthesia. The intranasal inoculation and bleeding in mice was performed after anaesthetizing the mice by inhalation of isofluorane in specialized chambers. All the efforts are made to minimize sufferings in both guinea pigs and mice.

All the experiments where 9-day old embryonated chicken eggs were used ended on or before day 13. Before collecting allantoic fluid from the eggs, the embryos were sacrificed by incubating the eggs at 4°C in a refrigerator for 2 hour.

### Cells, viruses, antibodies and protein

HEp-2, DF1, Vero and TZM-bl cells were grown in Dulbecco’s modified Eagle medium (DMEM) containing 10% fetal bovine serum (FBS). 293T/17 cells were grown and maintained in Opti-MEM I reduced serum medium containing 10% FBS. Recombinant and wild-type NDV strains were grown in 9-day-old specific-pathogen-free (SPF) embryonated chicken eggs. The modified vaccinia virus strain Ankara expressing the T7 RNA polymerase was grown in primary chicken embryo fibroblast cells. Purified recombinant HIV-1 BaL gp120 protein was obtained from the NIH AIDS Research and Reference Reagent Program (ARRRP). A pool of HIV gp120 monoclonal antibodies was kindly provided by Dr. Anthony DeVico, University of Maryland School of Medicine, UMB, Baltimore, MD.

### Construction of recombinant NDVs expressing HIV-1 gp140 and gp120 and gp160

A 2598-nucleotide (nt) cDNA encoding human-codon-optimized HIV-1 glycoprotein gp160 (852 amino acids [aa]) derived from the CCR5-tropic clade B strain BaL1 was modified by PCR to add NDV transcription signals and flanking PmeI sites and was inserted at the unique PmeI site between P and M genes in a cloned cDNA of the full-length antigenome of the lentogenic NDV vaccine strain LaSota (Figure 1) [27,28]. Additional constructs were made encoding two different versions of gp140, namely gp140L (2082 nt, 679 aa) and gp140S (2034 nt, 663 aa), as well as gp120 (1560 nt, 506 aa), and similarly were inserted at the PmeI site between the P and M genes (Figure 1). Recombinant viruses (designated rLaSota/gp160, rLaSota/gp140L, rLaSota/gp140S and rLaSota/gp120) were recovered as described previously [28] and were plaque purified and grown in 9-day-old embryonated SPF chicken eggs [29,30].

**Figure 1:** Gene map of recombinant NDV LaSota (rLaSota) and structures of gp160, gp120, gp140L, and gp140S. The proteins are shown as unprocessed primary translation products annotated to show the locations of the furin cleavage site, the membrane-proximal external region (MPER), the transmembrane (TM) and cytoplasmic (CT) domains, and the total aa lengths. The cDNAs encoding these proteins were modified by PCR to add NDV gene-start (GS) and gene-end (GE) transcription signals, an intergenic (IG) nucleotide, and flanking PmeI sites, and were inserted individually between the NDV P and M genes. Sequence flanking the Env ORFs is shown in positive-sense, and PmeI sites used in the construction are shown in italics. NDV genes (N, nucleoprotein; P, phosphoprotein; M, matrix protein; F, fusion glycoprotein; HN, hemagglutinin-neuraminidase protein; L, large polymerase protein) are shown as open boxes.

### Expression of HIV-1 gp140, gp120 and gp160 Env proteins in cells infected with recombinant virus

The expression of gp140, gp120 and gp160 by rLaSota/gp140L and rLaSota/gp140S, rLaSota/gp120 and rLaSota/gp160 was examined by Western blot analysis. Briefly, DF1 cells were infected with rLasota/gp140L, rLaSota/gp140S, rLaSota/gp120, rLaSota/gp160 and rLaSota at a multiplicity of infection (MOI) of 0.01 PFU. The cells were harvested at 48 h post-infection and lysed using radioimmunoprecipition buffer. The cell culture medium supernatants were collected at 48 h post-infection and were concentrated 10x by passing through Amicon filters. The cell lysate and cell culture medium supernatants were analyzed by Western blotting using a 1:10 dilution of a pool of gp120-specific monoclonal antibodies. Western blots were scanned and densitometric analysis of gp120 protein bands were performed by using the Photoshop program.

The expression of gp140, 120 and 160 by the recombinant viruses was further examined in Vero cells by immunofluorescence assay. Briefly, confluent monolayers of Vero cells on 4 well Lab-Tek chamber slides were infected with the recombinant viruses at an MOI of 0.1. After 24 h, the infected cells were washed with PBS and either fixed with 4% paraformaldehyde for 20 min at room temperature and permeabilized with 0.2% Triton X-100 in PBS for 10 min for detection of total antigen. After further washing with PBS, the cells were incubated for 30 min with 3% normal goat serum to block nonspecific binding sites and incubated for 1 h with 1:10 dilution of a pool of gp120-specific monoclonal antibodies. The cells were rinsed with PBS and incubated with a 1:1000 dilution of Alexa Fluor 488 conjugated goat anti-mouse immunoglobulin G antibody (Invitrogen, Carlsbad, CA) for 45 min. The cells were washed with PBS and analyzed with a fluorescent microscope.

### Analysis of HIV-1 gp160, gp140 and gp120 protein oligomers

The oligomeric state of gp140, gp120 and gp160 expressed by the NDV recombinants was analyzed by cross linking infected cell lysates followed by Western blotting. Briefly, lysates of rLaSota/gp140L, rLaSota/gp140S, rLasota/gp120, rLaSota/gp160 and rLaSota infected DF1 cells in PBS were incubated at room temperature for 30 min with a final concentration of 1 mM Dithiobis (succinimidyl propionate) [DSP; Pierce], a thiol-cleavable, amine-reactive and membrane-permeable crosslinker. After crosslinking, samples were prepared in Laemmli sample buffer (100 mM Tris, pH 6.8, 2% SDS, 15% glycerol) with or without 5% β- mercaptoethanol and boiled for 5 min to make reduced and non-reduced samples, respectively. SDS-PAGE and Western blot analysis were performed as described before.

### Pathogenicity of rNDVs in embryonated chicken eggs

The pathogenicity of rLasota/gp140L, rLasota/gp140S, rLasota/gp120, rLasota/gp160 and rLaSota in chickens was evaluated by an internationally established *in vivo* test: the mean death time (MDT) test in 9-day-old SPF embryonated chicken eggs. The MDT test was performed by a standard procedure [31]. Briefly, a series of 10-fold dilutions of fresh allantoic fluid from eggs infected with the test virus were made in sterile PBS, and 0.1 ml of each dilution was inoculated into the allantoic cavity of each of five eggs. The eggs were incubated at 37°C and examined four times daily for 7 days. The time that each embryo was first observed dead was recorded. The highest dilution that killed all embryos was considered the minimum lethal dose. The MDT was recorded as the time (in h) for the minimum lethal dose to kill the embryos. The MDT has been used to classify NDV strains as velogenic (MDT < 60 h), mesogenic (MDT 60 to 90 h), and lentogenic (MDT > 90 h).

### Growth characteristics of rNDVs in DF1 cells

To determine multicycle growth kinetics of rLaSota/gp140L, rLaSota/gp140S, rLaSota/gp120, rLaSota/gp160 and rLaSota, DF1 cells in duplicate wells of six-well plates were infected with each virus at an MOI of 0.01 PFU. After 1 h of adsorption, the cells were washed with DMEM and then incubated with DMEM containing 5% FBS and 5% allantoic fluid. The cell culture supernatant samples were collected and replaced with an equal volume of fresh medium at 8 h intervals until 64 h post-infection. The titers of virus in the samples were quantified by plaque assay in DF1 cells.

### Guinea pig immunizations

Female Hartley guinea pigs weighing approximately 375 gm each were obtained from Charles River Laboratories, Wilmington, MA. A total of 27 guinea pigs were divided into four groups of 6 animals each that received rLaSota/gp160, rLaSota/gp140L, rLaSota/gp140S, or rLaSota/gp120, and a control group of 3 animals that received the empty rLaSota vector. Animals were immunized by intranasal (i.n.) route on days 0 and 14 with 300 µl (150 µl in each nostril) of allantoic fluid containing 10^6^ PFU/ml of the indicated virus. All animals were sacrificed 76 days after the second boost (i.e. 90 days following the first immunization). Blood was collected on day 0 (pre-bleed) and on days 7, 14, 21, 28, 35, 42, 56, 70 and 90. Sera were prepared and stored at -70°C. Vaginal washes and fecal samples were collected in parallel with the blood samples. To collect vaginal washes, animal feeding needles (Fisher Scientific) were used to flush 100 µl of PBS containing protease inhibitor cocktail (Sigma) four to six times into vaginal cavity. Vaginal washes were spun at 10,000 rpm for 15 min to remove cellular debris and supernatants were collected and stored at -70°C. Fecal sample were collected in PBS containing antibiotics, vortexed and incubated at 37 °C for 20 min and spun at 4,000 rpm for 10 min. Supernatants were collected and stored at -70°C

### Measuring gp120-specific total IgG, IgG1, IgG2a and IgA antibodies in sera, vaginal washes and fecal samples by ELISA

HIV-1 Env-specific antibody titers were determined by isotype-specific ELISA. Ninety-six-well Maxisorp ELISA plates (Nunc, Denmark), coated overnight with 100 µl/well of 1 µg/ml purified recombinant HIV-1 BaL gp120 protein in sodium caronate/bicarbonate buffer (pH 9.8), were blocked first with 3% skimmed milk in water for 30 sec and then with 2% sucrose in water for 30 sec. Plates were dried for 2 h at 37°C. Serial dilutions of sera or vaginal washes or fecal samples from immunized guinea pigs were prepared in dilution buffer (Synbiotics Carporation, San Diego, CA), added to the plates, and incubated for 2 h at room temperature. The plates were washed three times with plate washing solution (Synbiotics Carporation) and incubated for 1 h with a 1:1,000 dilution of an isotype-specific secondary antibody; namely, horseradish peroxidase (HRP)-conjugated goat anti-guinea pig IgG (KPL, Gaithersburg, MD), goat anti-guinea pig IgG1, goat anti-guinea pig IgG2a (Novus Biologicals, Littleton, CO), or sheep anti-guinea pig IgA (Immunology Consultants Laboratory, Newberg, OR). The plates were washed three times and developed with ABTS (2,2'-Azinobis [3-ethylbenzothiazoline-6-sulfonic acid]-diammonium salt) peroxidase substrate solution (Synbiotics Corporation), stopped by the addition of peroxidase stop solution, and analyzed at 405 nm with ELx800 ELISA plate reader (BioTek, VT). ELISA endpoint titers were defined as the highest reciprocal serum dilution at which the mean OD value of duplicate wells were >2-fold above the mean OD value plus 2 SD of serum or vaginal wash or fecal sample from negative control animals. Commercial NDV ELISA kits (Synbiotics Corporation) was used to detect antibodies against the NDV antigens.

### Detection of Env-specific IFN-γ producing cells by intracellular cytokine staining (ICS)

Six-week-old female BALB/c mice (Charles River Laboratories, Wilmington, Massachusetts) in groups of six animals each were immunized by the i.n. route on days 0 and 14 with the indicated virus in 50 µl (25 µl in each nostril) of allantoic fluid containing 10^5^ PFU/ml. Splenocytes were collected on day 56 and stimulated for 12 h with either 10 µg/ml of HIV-1 consensus subtype B 10-mer overlapping Env peptide pools (AIDS Research and Reference Reagent Program) or medium alone. Cells were incubated for 6 h with 10 µg/ml brefeldin A (Sigma). After blocking Fcγ receptors (rat anti-mouse CD16/32; BD Biosciences), cells were stained with Alexa Fluor 488-conjugated anti-mouseCD3ε and APC-Cy™7 conjugated anti-CD4 and per CP-Cy ^TM^5 conjugated anti-mouse CD8 for 30 min at 4°C. The cells were fixed, permeabilized (Cytofix/Cytoperm Plus, BD Biosciences) and stained with PE anti–IFN-γ mAbs for 30 min at 4°C (BD Biosciences). Cells were analyzed by flow cytometry and Flowjo software was used for data analysis. The frequencies of cells positive for IFN-γ+ and CD4 or CD8 were determined. Data are representative of three experiments where spleens from two mice were pooled in each experiment.

### Neutralization assays

Neutralizing antibody activity was measured in 96-well culture plates by using Tat-regulated Luc reporter gene expression to quantify reductions in virus infection in either TZM-bl or A3R5.7 cells. Assays in TZM-bl cells were performed with HIV Env-pseudotyped viruses as described previously [32]. TZM-bl cells were used for neutralization of clade B tier 1 HIV-1 strains BaL.26 and MN.3 and heterologous clade B tier 2 HIV-1 strains RHPA4259.7 and TRO.11. Briefly, neutralization assays were performed with serial dilutions of heat-inactivated (56°C, 1 hr) samples. Serum samples were diluted over a range of 1:20 to 1:43740 in cell culture medium and were pre-incubated with virus (~150,000 relative light unit equivalents) for 1 hr at 37 °C before addition of cells. Following 48 hr incubation, cells were lysed and luciferase activity was determined using a microtiter plate luminometer and BriteLite Plus Reagent (PerkinElmer). The A3R5.7 cell line (A3.01/R5.7) is a derivative of the CEM human lymphoblastoid cell line that naturally expresses CD4 and CXCR4 [33] and was engineered to express CCR5 [34]. The A3R5 assay was performed with clade B tier 2 HIV-1 strains SC22.3C2.LucR. T2A.ecto and REJO. LucR. T2A.ecto essentially as previously described [35]. As with the TZM-bl assay, diluted samples were incubated with virus (~50,000 RLU equivalents) for 1 hr at 37 °C prior to adding cells. After incubating for 4 days, a defined portion of the cell suspension was transferred to 96-well white solid plates (Costar) for measurement of luminescence using the ViviRen Live Cell Substrate as described by the supplier (Promega). For both the TZM-bl and A3R5 assays, neutralization titers are the sample dilution at which relative luminescence units (RLU) were reduced by 50% compared to RLU in virus control wells after subtraction of background RLU in cell control wells. For each animal in this study, pre- and post-immune serum samples were assayed side-by-side. As is often the case with guinea pig sera, a low-level background signal was present in many pre-immune serum samples; the background has been subtracted from the neutralization titers presented.

### Statistical analysis

Statistical analysis of serological responses was performed by unpaired t test (two-tailed) with the use of Prism 5.0 (Graph Pad Software Inc., SanDiego, CA) with a significance level of *P* <0.05.

## Results

### Generation of rNDVs expressing HIV-1 gp160, gp140L, gp140S, and gp120

A recombinant version of the avirulent NDV vaccine strain LaSota was used to construct four viruses expressing different forms of the Env glycoprotein of HIV-1 strain BaL.1, namely: (i) the full-length, 852-aa gp160 protein (virus rLaSota/gp160); (ii) a 679-aa gp140 protein (gp140L, virus rLaSota/gp140L) that contained the complete 30-aa MPER at its C-terminus and terminated with the sequence WYIKI immediately adjacent to the transmembrane domain; (iii) a shorter, 663-aa gp140 protein (gp140S, virus rLaSota/gp140S) that contained a partial, 14-aa long MPER at its C-terminus and terminated with the sequence DKWAS; and (iv) a 560-aa gp120 protein (virus rLaSota/gp120) that terminated with the cleavage site sequence REKR (Figure 1). The recombinant viruses were recovered and propagated in embryonated chicken eggs with peak titers of 10^8^ to 10^9^ HA units and in DF1 cells with peak titers 10^7^ to 10^8^ pfu/ml. To determine the stability of the gp160, gp140 and gp120 genes in rLaSota vector, the recovered viruses were passaged 10 times in embryonated chicken eggs and the sequences were confirmed.

### Expression of HIV-1 gp140 and gp120 and gp160 Env proteins and analysis of oligomers

To investigate the expression of the various forms of Env, DF1 cells were infected with rLaSota/160, rLaSota/gp140L, rLaSota/gp140S, and rLaSota/gp120, and cell lysates and culture medium supernatants were harvested, subjected to gel electrophoresis, and analyzed by Western blot using a pool of gp120-specific monoclonal antibodies. Analysis of cell lystates revealed the presence **of** precursor protein (either 160 kDa or 140 kDa) as well as the 120 kDa protein derived by cleavage of gp140 or gp160 or expressed directly by rLaSota/gp120 (Figure 2A). Densitometric analysis of Western blot showed that level of gp140 and gp120 proteins expressed by rLaSota/gp140S was 2-fold higher compared to rLaSota/gp140L (Figure 2A). Analysis of medium supernatants showed that gp120 was secreted from cells infected with rLaSota/gp140L, rLaSota/gp140S, and rLaSota/gp120, whereas gp120 expressed by rLaSota/gp160 remained cell-associated (Figure 2B). Densitometric analysis of gp120 protein band present in Western blot revealed that the level of gp120 secreted by rLaSota/gp140S was 3-fold higher compared to rLaSota/gp140L. The intracellular expression of Env protein in response to the NDV vectors also was analyzed in Vero cells by indirect immunofluorescence using a pool of gp120-specific monoclonal antibodies (Figure 3). This showed that the distribution of Env protein expressed by rLaSota/gp140L, rLaSota/gp140S, and rLaSota/gp120 was quite different compared to rLaSota/gp160, which is not surprising since the substantial secretion of gp120 observed with the first three viruses would involve the secretory pathway, whereas, in contrast, Env protein expressed by rLaSota/gp160 remained cell-associated and would accumulate on the plasma membrane.

**Figure 2:** Detection of NDV-expressed Env proteins present in infected-cell lysates (A) and the cell culture medium (B). DF1 cells were infected with indicated viruses at an MOI of 0.01 PFU. After 48 h, the cell culture medium supernatants and cells were collected and processed. (A) The cell lysates were prepared from cells and subjected to SDS-PAGE under reducing conditions. (B) The cell culture medium supernatants were concentrated 10x by passing through Amicon filters and subjected to SDS-PAGE under reducing conditions. The gels were analyzed by Western blotting using a pool of gp120-specific monoclonal antibodies. The positions of HIV-1 gp160, gp140 precursor gp120 are indicated by arrows in the right margin. Molecular masses of marker proteins (in kilodaltons) are shown in the left margin.

**Figure 3:** Immunofluorescence of Env protein expressed in Vero cells infected with rLaSota/gp160 (panel a), rLaSota/gp140L (panel b), rLaSota/gp140S (panel c), rLaSota/gp120 (panel d) and rLaSota (panel e) at an MOI of 0.1 PFU. Twenty-four h post-infection, the infected cells were fixed with paraformadehyde and permeabilized with Triton X-100 for detection of total antigen inside the cell. The cells were probed with a pool of gp120-specific monoclonal antibodies followed by incubation with Alexa Fluor 488-conjugated goat anti-mouse IgG antibodies, and analyzed by immunofluorescence. The cells were visualized under Nikon Eclipse TE fluorescent microscope. Arrows indicate areas of positive immunofluorescence.

The oligomeric state of the Env proteins in DF1 cells infected with rLaSota/gp140L, rLaSota/gp140S, rLaSota/gp120, and rLaSota/gp160 was investigated by preparing infected cell lysates and subjecting them to cross-linking with the thiol-cleavable cross-linker DSP, followed by SDS-PAGE under reducing and non-reducing conditions and immunoblotting with gp120-specific monoclonal antibodies (Figure 4). Cross-linked Env protein expressed by rLaSota/gp160 migrated under non-reducing conditions as a broad oligomeric band of molecular mass greater than 188 kDa, as we previously described [27]. Under non-reducing conditions, cross-linked Env protein expressed by rLasota/gp140S migrated as a diffuse band of higher molecular weight, corresponding to higher order oligomeric forms. Unexpectedly, very little Env protein oligomers could be detected in rLasota/gp140L-infected cells. The bulk of cross-linked gp120 expressed by rLaSota gp120 migrated under non-reducing conditions as higher order oligomers. These data suggest that rLaSota/gp140S and rLaSota/gp120, similar to rLaSota/gp160, support the expression of one predominant oligomeric species of molecular mass greater than 188 kDa, probably representing dimers and or trimers.

**Figure 4:** Oligomeric status of NDV-expressed Env proteins. DF1 cells were infected with indicated viruses at an MOI of 0.01 PFU. After 48 h, the cells were collected and cross-linked with DSP and subjected to SDS-PAGE under reducing (+R) or non-reducing (-R) conditions. The gels were analyzed by Western blotting using a pool of gp120-specific monoclonal antibodies. The positions of HIV-1 gp160, gp140 precursor gp120 are indicated by arrows in the right margin. Molecular masses of marker proteins (in kilodaltons) are shown in the left margin.

### Biological characterization of rNDVs expressing gp140, 120 and 160 proteins

The multicycle growth kinetics of rLaSota/gp140L, rLaSota/gp140S rLaSota/gp120, rLaSota/gp160 in DF1 cells showed that the replication of these recombinants was essentially indistinguishable from that of parental rLaSota virus (Figure 5). The pathogenicity of these recombinants and their parental rLaSota virus was evaluated in 9-day-old embryonated chicken eggs by the MDT (mean death time) test. The values of MDT for rLaSota, rLaSota/gp140L, rLaSota/gp140S, rLaSota/gp120 and rLaSota/gp160 were 105 h, 107 h, 107 h, 106 h and 109 h, respectively. This showed that the insertion of the foreign gene conferred a marginal amount of attenuation to the NDV vector.

**Figure 5:** Comparison of multicycle growth kinetics of rLaSota/gp160 (panel A), rLaSota/gp140L (panel B), rLaSota/gp140S (panel C), rLaSota/gp120 (panel D) viruses, each compared with the empty vector rLaSota virus. DF1 cells were infected with each virus at an MOI of 0.01 and cell culture media supernatant aliquots were harvested at 8 h intervals until 64 h post-infection. The virus titers in the aliquots were determined by plaque assay in DF1 cells. Values are averages from three independent experiments.

### Infection of guinea pigs

To evaluate the immunogenicity of Env protein expressed by the various NDV recombinants, we immunized outbred female Hartley guinea pigs (n=6 for groups immunized with rLaSota/gp140L, rLaSota/gp140S, rLaSota/gp120 and rLaSota/gp160 and n=3 for the empty vector rLaSota control) on days 0 and 14 (Figure 6). Each animal received a dose of 300 µl (150 µl in each nostril) of allantoic fluid containing 10^6^ PFU/ml of recombinant virus. We chose the i.n. route because it elicited the highest immune responses in our previous study with rNDV expressing gp160 protein [27]. The animals did not show any overt clinical signs of infection or any loss of body weight throughout the study. However, three animals each from the rLaSota/gp160 and rLaSota/gp140L groups and one animal from the rLaSota/gp120 group died due to physical injury (bone fracture) during captivity that was unrelated to the immunizations. Post-mortem analysis of different tissues such as lungs, trachea, spleen and brain revealed no lesions and no virus was isolated from these tissues.

**Figure 6:** Immunization schedules. A. Guinea pig immunization. Twenty seven guinea pigs were divided into 5 groups (n=6 for rLaSota/gp160, rLaSota/gp140L, rLaSota/gp140S, rLaSota/gp120 groups; n=3 for rLaSota group). Animals in each group were immunized with two doses of each recombinant virus on days 0 and 14 by i.n. route of administration. Each dose consisted of 300 µl (150 µl in each nostril) of allantoic fluid containing 10^6^ PFU/ml of virus. Blood, vaginal washes and fecal samples were collected on days 0, 7, 14, 21, 28, 42, 56, 70 and 90. All animals were sacrificed on day 90. B. Mice immunization. Thirty mice were divided in to 5 groups (n=6/group). Animals in each group were immunized with two doses of virus on days 0 and 14 by the i.n. route of administration. Each dose consisted of 50 µl (25 µl in each nostril) of allantoic fluid containing 10^5^ PFU/ml of virus. All animals were sacrificed on day 56 and splenocytes were collected.

### Humoral immune responses

The induction of NDV-specific serum antibodies was measured on days 28 and 56 using an NDV-specific ELISA (Figure 7A). All four animal groups exhibited high levels of NDV-specific IgG antibodies on these days, suggesting that each of the viruses replicated to same extent in the immunized animals.

**Figure 7:** NDV-specific total IgG (panel A), and HIV-1 gp120-specific total IgG (panel B), IgG1 (panel C) and IgG2 (panel D) responses in guinea pig sera. The guinea pigs were immunized with the indicated rNDVs by the i.n. route. (A) The guinea pig sera were analyzed for NDV-specific antibodies by commercial NDV ELISA kits (Synbiotics Corporation). Mean ELISA end-point titers of NDV-specific serum antibodies on days 28 and 56 are shown. (B-D) The guine pig sera were analyzed by HIV-1 gp120 specific total IgG, IgG1 and IgG2 antibodies by isotype-specific ELISA with purified gp120. Mean ELISA end-point titers of gp120-binding serum antibodies of the indicated isotype on days 0, 7, 14, 21, 28, 42, 56, 70 and 90 are shown. Antibodies specific to gp120 were not detected in any animal on any day in the control rLaSota group. The graph shows the geometric mean value ± SEM for 3 animals in rLaSota, rLaSota/gp160 and rLaSota/gp140L groups, 6 animals in rLaSota/gp140S group and 5 animals in rLaSota/gp120 group. Arrows indicate time of rNDV immunizations on days 0 and 14. Statistical differences between the groups were calculated by unpaired t test (two-tailed). 1* indicates statistically significant differences (*P*<0.05) of rLaSota/gp140S vs. rLaSota/gp160, rLaSota/gp140L and rLaSota/gp120 groups. 2* indicates statistically significant differences (*P*<0.05) of rLaSota/gp140S vs. rLaSota/gp160 and rLaSota/gp140L groups.

The induction of HIV-1 Env-specific serum antibodies was measured on days 7, 14, 21, 28, 42, 56, 70 and 90. Total serum IgG specific to BaL.1 gp120 was measured at each time point by ELISA (Figure 7B). Responses were detected on day 21 following the initial immunization in all of the groups. The boost on day 14 was followed by increased immune responses in all the groups. The highest gp120-spectific total IgG titer was observed with the rLaSota/gp140S group, followed by the rLasota/gp160 and rLaSota/gp120 groups, and the lowest titer was observed with rLaSota/140L. On day 42, rLaSota/gp140S group showed significantly higher titer compared to all the other groups (*P*<0.0001 for gp140S versus gp160 and gp40L groups, *P*=0.0008 for gp140S versus gp120 group) and on day 56, it showed significantly higher titer compared to rLaSota/gp160 and rLaSota/gp140L groups (*P*<0.05).

In addition, serum IgG1 and IgG2a responses specific to BaL.1 gp120 were measured by isotype-specific ELISA (Figure 7C and D). Responses were detected on day 21 after the first immunization in all of the groups, and responses peaked by day 42. The IgG1 response was strongest in rLaSota/gp140S group followed by rLaSota/gp120, rLaSota/gp140L and rLaSota/gp160 groups. On day 42, rLaSota/gp140S group showed significantly higher titer compared to all the other groups (*P*<0.05), whereas on days 28, 56, 70 and 90, the IgG1 titer induced by rLaSota/gp140S was significantly higher compared to rLaSota/gp160 and rLaSota/gp140L (*P*<0.05). The IgG2 response also was strongest in rLaSota/gp140S group followed by rLaSota/gp120, rLaSota/gp160, and rLaSota/gp140L. On days 28 and 42, the IgG2 response induced by rLaSota/gp140S was significantly higher compared to rLaSota/gp160 and rLaSota/gp140L (*P*<0.05). We also calculated the ratio of serum IgG1:IgG2a to assess the Th1/Th2 balance. The ratio for rLaSota/gp160 was 1:3 on day 28 and 1:8 on day 90, indicative of a Th1-biased response. In contrast, the ratios for rLaSota/gp140L, rLaSota/gp140S, and rLaSota/gp120 varied from 1:0.7 to 1:1.4 on days 28 to 90 post-immunization and thus showed mixed Th1/Th2 responses. In addition, we assayed gp120-specific serum IgA in all the groups, but all animals at all-time points were negative.

### Mucosal immune responses

Vaginal washes were collected from each animal at each time point and evaluated by ELISA using BaL.1 gp120-coated plates (Figure 8). In all the groups, the titer of total IgG peaked on day 42, decreased by day 56-70, and surprisingly peaked again on day 90 (Figure 8A). The response was greatest in the rLaSota/gp140S group followed by rLaSota/gp120, rLaSota/gp160, and rLaSota/gp140L. On day 56, the response induced by rLaSota/gp140S was significantly higher compared to rLaSota/gp160 and rLaSota/gp140L (*P*<0.05). We assayed the total IgG response in fecal samples in all of the groups but unable to detect any titer. We also analyzed the IgG1 and IgG2a responses in vaginal washes in all the groups (Figure 8B and C). Similar to total vaginal IgG response, the IgG1 and IgG2a responses peaked on day 42, decreased on day 56-70 and increased on day 90. The IgG1and IgG2a responses were strongest with rLaSota/gp140S followed by rLaSota/gp20, rLaSota/gp160, and rLaSota/gp140L. On day 42, the IgG1 response induced in rLaSota/gp140S group was significantly higher compared to rLaSota/gp160 rLaSota/gp140L groups (*P*<0.05), whereas on day 56, it was significantly higher in this group compared to all the other groups (*P*<0.05). Also the IgG2a response induced on day 56 in rLaSota/gp140S group was significantly higher compared to rLaSota/gp160 and rLaSota/gp140L groups (*P*<0.05). The vaginal IgG1:IgG2a ratio varied from 1: 3 to 1:7 at different time points for the rLaSota/gp160 group, indicative of a Th1-biased response. In the other groups, the vaginal Th1:Th2a ratio varied at different time points from 1:0.7 to 1:4.5, 1:0.6 to 1:2.3 and 1:1 to 1:4 for rLaSota/gp140L, rLaSota/gp140S, and rLaSota/gp120, indicative of a mixed Th1/Th2a response. BaL.1 gp120-specific IgA responses in vaginal washes also were measured (Figure 8D). A low titer was detected in the all the groups. The titer peaked on day 42, dropped on day 56 and increased slightly on day 90. The strongest response was detected in the rLaSota/gp140S group, followed by rLaSota/gp160, rLaSota/gp120, and rLaSota/gp140L.

**Figure 8:** HIV-1 gp120-specific total IgG (panel A), IgG1 (panel B), IgG2a (panel C) and IgA (panel D) antibodies in vaginal washes collected from guinea pigs, detected by isotype-specific ELISA with purified gp120. The guinea pigs were immunized with the indicated rNDVs by the i.n. route. Mean ELISA end-point titers of gp120-binding vaginal wash antibodies of the indicated isotype on days 0, 7, 14, 21, 28, 42, 56, 70 and 90 are shown. Antibodies specific to gp120 were not detected in any animal on any day in control rLaSota group. The graph shows the geometric mean value ± SEM for 3 animals in rLaSota, rLaSota/gp160 and rLaSota/gp140L groups, 6 animals in rLaSota/gp140S group and 5 animals in rLaSota/gp120 group. Arrows indicate time of rNDV immunizations on days 0 and 14. Statistical differences between the groups were calculated by unpaired t test (two-tailed). 1* indicates statistically significant differences (*P*<0.05) of rLaSota/gp140S vs. rLaSota/gp160, rLaSota/gp140L and rLaSota/gp120 groups. 2* indicates statistically significant differences (*P*<0.05) of rLaSota/gp140S vs. rLaSota/gp160 and rLaSota/gp140L groups.

### Neutralizing antibody (NAb) responses

Sera from days 28, 56, 70 and 90 from animals immunized with the rNDVs expressing gp140, gp120 and gp160 were evaluated in the TZM bl assay (which assays HIV-1 infection by measuring Tat-regulated luciferase expression in an indicator cell line) for the ability to neutralize homologous clade B tier 1 HIV-1 strains BaL.26 and MN.3 and heterologous clade B tier 2 HIV-1 strains RHPA4259.7 and TRO.11. NAb activity (expressed as IC_50_ value) against HIV-1 strain Bal.26 was detected in sera from all of the animals immunized with NDV expressing the various Env-derived proteins, with the highest titer observed with rLaSota/gp140S followed by rLaSota/gp120, rLaSota/gp160, and rLaSota/gp140L (Figure 9A). On days 28, 56, 70 and 90, the mean IC_50_ titers induced by rLaSota/gp140S was higher than rLaSota/gp160 and rLaSota/gp140L but it was significantly higher particularly on days 28 and 70 (*P*<0.05). Compared to rLaSota/gp120 group, NAb activity induced in rLaSota/gp140S group was also higher on all the days but it was significantly higher on day 28 (*P* = 0.002). A comparison of mean IC_50_ titres against HIV-1 strain MN.3 among all the groups on days 28 and 56 showed a significantly stronger NAb responses in rLaSota/gp140S group (*P*<0.05) [Figure 9B]. On day 70, NAb response was also significantly stronger in rLaSota/gp140S group compared to rLaSota/gp160 and rLaSota/gp140L groups. These data indicated that NAb response induced by rLaSota/gp140S against homologous clade B tier 1 HIV-1 strains BaL.26 and MN.3 was significantly stronger compared to other recombinant viruses early on but the differences diminished over time particularly for BaL.26 strain. Further, analysis of sera of day 56 of all the groups indicated a weak neutralization response against the clade B tier 2 viruses RHPA4259.7 and TRO.11 in TZM bl assay (Figure 9C). We then used more sensitive A3R5 assay to look for neutralization of Clade B tier 2 HIV-1 strains SC22.3C2.LucR. T2A.ecto and REJO. LucR. T2A.ecto. As shown in Figure 9C, NAb activity induced against SC22.3C2.LucR. T2A.ecto by rLaSota/gp140S was higher compared to other groups and was significantly greater compared to rLaSota/gp140L and rLaSota/gp120 groups (*P*<0.05). No response was observed against REJO. LucR. T2A.ecto virus (data not shown).

**Figure 9:** Virus neutralizing antibody activity (50%-inhibitory-concentration [IC_50_] titers) against homologous HIV-1 clade B tier 1 strains (BaL.26 and MN.3) and heterologous clade B tier 2 strains (RHPA4257.7, TRO.11, and SC22.3C2.LucR. T2A.ecto) in sera from guinea pigs immunized with the indicated rNDVs. (A) Guinea pig sera obtained on days 28, 56, 70 and 90 were tested against BaL.26 pseudovirus by the TZM-bl assay (B) Guinea pig sera obtained on days 28, 56, 70 and 90 were tested against MN.3 pseudovirus by the TZM-bl assay (C) Guinea pig sera obtained on day 56 were tested against RHPA4257.7 and TRO.11 by the TZM-bl assay, and against SC22.3C2.LucR. T2A.ecto by the A3R5 assay. Horizontal bars indicate the geometric mean titer. Pre-immune sera were used to establish baseline-neutralizing activity in each individual guinea pig, and these values were subtracted from the values shown. The neutralizing antibody activity against each virus in sera obtained from guinea pigs immunized with rLaSota virus was <20. Statistical differences between the groups were calculated by unpaired t test (two-tailed) and shown by the numbers underneath the horizontal line. * indicates statistically significant differences (*P*<0.05) between groups.

### Cellular Immune Responses

The ability of rNDVs to stimulate cellular immune responses against HIV-1 Env was evaluated in female BALB/c mice (n=6/group). This model was used because of the availability of immunological reagents. Mice were inoculated i.n. on days 0 and 14 with the various rNDVs expressing gp140S, gp140L, gp120 and gp160, and on day 56 splenocytes were isolated (Figure 6B). The splenocytes were stimulated in vitro with Env peptides, and processed for intracellular cytokine staining of IFN-γ and staining for CD4 or CD8 (Figure 10). A significant number of IFN-γ-producing CD4^+^ T cells and CD8^+^ T cells were detected, and were higher in the mice that received rLaSota/gp140S and rLaSota/gp120 than for rLaSota/gp160 and rLaSota/gp140L. Mice immunized with rLaSota/gp140S and rLaSota/gp120 demonstrated 9- and 5- fold increases in IFN-γ+CD4+ T cells compared to rLaSota/gp160 (Figure 10A). The number of IFN-γ+CD8+ T cells was higher with rLaSota/gp120, rLaSota/gp140S and rLaSota/gp140L compared to rLaSota/gp160 (Figure 10B) Collectively, these results demonstrate that administration of rNDV expressing gp140S can induce robust CD4+ and CD8+ T cell responses in addition to humoral and mucosal immune responses.

**Figure 10:** HIV-1 Env-specific CD4+ (panel A) and CD8+ (panel B) T cell response. Mice in groups of 6 were immunized with 10^5^ PFU/ml of the indicated rNDV by the i.n. route on days 0 and 14. On day 56, splenocytes were isolated, stimulated with a pool of overlapping Env peptides, and processed for intracellular cytokine staining for IFN-γ and CD4 and CD8.

## Discussion

Recently, the modest success of the recent phase III RV144 trial, employing a prime-boost vaccine regime with a recombinant canarypox vector and purified recombinant gp120, emphasized that Env-based immunogens are important HIV-1 vaccine candidates [36]. It is important to further explore the immunogenicity of different structural variants of the Env glycoprotein. In addition, the optimal means to present Env antigen to the immune system requires continued investigation, particularly presentation by live viral vectors. Different Env-based immunogens including gp120 and gp140 have been shown to induce variable humoral and CTL responses in animal models. The results of clinical trials indicated that soluble gp120 elicits antibodies of narrow neutralization specificities that are unable to neutralize primary isolates [37-39]. A critical deficiency of gp120 vaccines is the absence of epitopes that are present in relatively conserved gp41 regions such as MPER. Therefore, gp160 was considered to be a better immunogen than gp120. A previous study showed that gp160 is cytotoxic but that truncation of its C-terminus to 140 kDa, by removal of the transmembrane and cytoplasmic domains, could remove its cytotoxicity [40]. Thereafter, more attention has been focused on generation of versions such as gp140 because it contains the entire ectodomain of HIV-1 Env, has the potential to form trimers indicative of an intact authentic conformation, and can be secreted from expressing cells. To stabilize recombinant gp140 trimers and to elicit a better immune response against HIV-1, various strategies have been employed, such as engineering a cleavage-deficient form produced by deletion of the furin cleavage site, or introduction of disulfide bonds to covalently link gp120 and gp41, or incorporation of trimerization motifs into the gp41 ectodomain [11]. In the present study, we used a live, replication-competent NDV vector to express and compare several forms of Env. Each Env ORF was engineered to be under the control of NDV transcription signals in the NDV genome and to be expressed as a separate mRNA. This strategy would provide for de novo synthesis of correctly folded and processed trimers in vivo. We retained the furin cleavage site on the premise that native cleavage might be important to the correct conformation. We generated two forms of 140, namely gp140L and gp140S that contained complete or partial MPER, respectively, and compared these to gp120 and gp160. The NDV vector was based on the LaSota strain, which is a naturally-occurring avirulent strain that is commonly used as a live NDV vaccine in chickens and thus poses no agricultural concerns.

Initially, we investigated whether rNDV could efficiently express correctly folded gp140 and gp120 molecules and whether these molecules could be cleaved, assemble to form oligomers, and be secreted. NDV-expressed gp160, gp140L, and gp140S were shown to be cleaved, although cleavage of gp140L was somewhat less efficient. NDV-expressed gp120 and gp140S were efficiently secreted, whereas secretion of gp140L was much less efficient, and gp160 was not secreted consistent with its membrane-bound status. Chemical cross-linking and gel electrophoresis showed that gp160, gp140S, and gp120 efficiently formed conformationally intact higher-order oligomers, whereas gp140L did not. The low level of expression, cleavage, oligomer formation, and secretion by gp140L suggested that either this truncation mutant might have a defect in folding or the protein produced by this mutant could be unstable and rapidly degraded.

Previously, we have shown the potential of rNDV as a vaccine vector to deliver HIV-1 gp160 protein by the i.n. route in guinea pigs [27]. In the present study, we immunized guinea pigs with two doses of the various NDV constructs by the i.n. route and evaluated the resulting serum and mucosal antibodies for the ability to bind to purified gp120 in ELISA and to neutralize homologous and heterologous strains of HIV-1. Our results showed that the rLaSota/gp140S group exhibited higher humoral and mucosal immune responses compared with the other groups. In addition, the immune responses elicited by rLaSota/140S and rLaSota/120 groups were qualitatively different in terms of antibody isotypes compared to responses elicited by rLaSota/160 group. Whereas, similar to our previous studies, rLaSota/160 induced a Th1-biased response (lower IgG1:IgG2a ratio), rLaSota/gp140S and rLaSota/120 induced mixed Th1/Th2 responses (higher IgG1:IgG2a ratio). Further, the neutralization responses elicited against the homologous strain BaL.26 and the laboratory adapted heterologous strain MN.3 differed among the various constructs and showed the following rank order: rLaSota/140S>rLaSota120>rLaSota160 >rLaSota140L. The lower IgG1 and neutralizing antibody responses for rLaSota/gp160 compared to rLaSota/gp140S and rLaSota/gp120 could be due to several reason: i) the transmembrane and cytoplasmic domains present in gp160 might influence the conformation of gp120, ii) some non-neutralization epitopes might be present on these domains, and the immune responses generated against these epitopes might create hindrance to neutralizing antibodies, iii) previous studies indicated that the cytoplasmic domain of gp41 contains some down regulatory sequences that could affect cell surface expression of gp160 [41,42], and (iv) the ability of gp140S and gp120 to be both cell-associated and secreted may provide increased immunogenicity. The finding that the immune responses elicited by NDV-expressed gp140S was superior to that of gp120 and gp160 supports the concept that trimeric gp140 envelope glycoprotein in a soluble form is a more efficient Env immunogen [43-46].

In the present study, we found that immunization of guinea pigs and mice with rLaSota/gp140L resulted in humoral, mucosal and cellular immune responses that are lower than those induced by rLaSota/gp140S. The gp41 sequence of rLaSota/gp140L is 16 aa longer and contains the complete 30-aa long MPER compared to shorter MPER sequence of gp41 present in rLaSota/gp140S. The lower level of immunogenicity induced by rLaSota/gp140L compared to rLaSota/gp140S could be due to a lower level of gp140L expression, inefficient cleavage, oligomerization or secretion. It is also possible that the presence of complete C-terminal MPER region in gp140L exerted immune suppression due to mimicry of this region to the self-protein cardiolipin [47]. It was shown earlier that the MPER region is weakly immunogenic when it was presented to the immune system on particulate Hepatititis B surface antigen particles [48]. However, recently analysis of human monoclonal antibody 10E8, isolated from an HIV-1 infected individual with high neutralization titers, demonstrated that the breadth of neutralizing antibody response of this antibody is mediated by recognition of MPER [49]. The differences in the immunogenicity between rLaSota/gp140L and rLaSota/gp140S warrant further investigation.

We have demonstrated that rNDV expressing HIV Env protein is able to induce a potent humoral immune response against HIV [27]. However, several studies including recently concluded RV144 trial in Thailand suggested that in addition to Env specific antibodies, CD4+ T cell response are important for protection against HIV-1 [36,50]. Studies in Elite controller and in macaque models indicated that in addition to CD4+ T cells, CD8+ T cells appear to play a key role in control of viral replication and level of set point viral load [51-53] Little information is available regarding the induction of T cell responses against foreign proteins expressed by NDV-based vectors. In this study we evaluated rNDV expressing HIV Env proteins to induce HIV-1 specific CD4+ and CD8+ T cells in mice. Inoculation of mice with rNDV expressing different forms of HIV Env resulted in both CD4+ and CD8+ T cell immune responses against HIV Env. rLaSota/gp140S and rLaSota/gp120 produced higher T cell responses compared to other recombinants. These results have indicated that NDV is promising vector for inducing T cell responses against HIV Env.

A major limitation of virus-based vectors is interference by anti-vector antibodies [54,55]. As noted, NDV has the advantage of being antigenically distinct from other common human pathogens, and thus its use should be unaffected by antibodies commonly present in the human population. Vector-specific antibodies also arise following the first vaccine administration, and these may interfere with a subsequent application of the same vaccine [56]. However, in the present study we found that NDV vectors can elevate the level of humoral and mucosal responses to the transgene following a booster vaccination. We think that NDV can re-infect because its low level of replication does not allow for the induction of solid immunity after only one inoculation. It also is possible that NDV is unusually immunogenic as it is a potent inducer of interferon and dendritic cell maturation and so even a low level of replication is very immunogenic. There was a decrease in IgG titer in vaginal washes on day 56 or 70 and surprisingly, it increased again on day 90. A possible explanation for this increase could be the production of long lived plasma cells from bone marrow [57].

In summary, we evaluated the potential of NDV strain LaSota as a vaccine vector for expressing different forms of the HIV-1 Env protein. In particular, we compared the humoral and mucosal immune responses in guinea pigs and cellular immune responses in mice induced by rNDVs expressing gp140S, gp140L, gp120 and gp160. Our results showed that rNDV is a promising vector that can induce mucosal, humoral and cellular immune responses against HIV-1 Env proteins. We evaluated two forms of gp140 expressed by rNDV and, surprisingly, found that deletion of part of MPER resulted in increased immunogenicity. The immune responses elicited by gp140S oligomers expressed by rNDV were several fold higher compared to those induced by rNDVs expressing gp120 and gp160 oligomers. Further, the ability of rLaSota/gp140S to induce neutralizing antibody responses against homologous BaL.26 and laboratory adapted MN.3 was superior to rLaSota/gp120 and rLaSota/gp160. We conclude that rNDV expressing soluble gp140 oligomers lacking the complete MPER produces strong mucosal, humoral and cellular immune responses that warrants further investigation in nonhuman primates.
